The article "Roles of the PI3K/AKT/mTOR signalling pathways in neurodegenerative diseases and tumours" was retracted in 2021. Reason: plagiarism.

# Roles of the PI3K/AKT/mTOR signalling pathways in neurodegenerative diseases and tumours

**DOI:** 10.1186/s13578-020-00416-0

**Published:** 2020-04-01

**Authors:** Fei Xu, Lixin Na, Yanfei Li, Linjun Chen

**Affiliations:** 1 Department of Microbiology and Immunology, Shanghai University of Medicine & Health Sciences, 279 Zhouzhu Rd, Shanghai, 201318 China; 2 Collaborative Innovation Center of Shanghai University of Medicine & Health Sciences, Shanghai, 201318 China; 3 Department of Inspection and Quarantine, Shanghai University of Medicine & Health Sciences, Shanghai, 201318 China

**Keywords:** PI3K/AKT/mTOR signalling pathway, Regulatory mechanism, Ischaemic brain injury, Neurodegenerative diseases, Tumour

## Abstract

The PI3 K/AKT/mTOR signalling pathway plays an important role in the regulation of signal transduction and biological processes such as cell proliferation, apoptosis, metabolism and angiogenesis. Compared with those of other signalling pathways, the components of the PI3K/AKT/mTOR signalling pathway are complicated. The regulatory mechanisms and biological functions of the PI3K/AKT/mTOR signalling pathway are important in many human diseases, including ischaemic brain injury, neurodegenerative diseases, and tumours. PI3K/AKT/mTOR signalling pathway inhibitors include single-component and dual inhibitors. Numerous PI3K inhibitors have exhibited good results in preclinical studies, and some have been clinically tested in haematologic malignancies and solid tumours. In this review, we briefly summarize the results of research on the PI3K/AKT/mTOR pathway and discuss the structural composition, activation, communication processes, regulatory mechanisms and biological functions of the PI3K/AKT/mTOR signalling pathway in the pathogenesis of neurodegenerative diseases and tumours.

## Key points

1. We summarize the PI3K/AKT/mTOR signalling pathway and its composition.
2. We list the current commonly PI3K/AKT/mTOR inhibitors for preclinical and clinical development.
3. We summarize the recent research progress regarding the PI3K/AKT/mTOR signalling pathway in common human diseases (neurodegenerative diseases and tumours).
4. We aimed to provide useful suggestions for additional research on the mechanism underlying the biological regulation of this pathway.

## Introduction

Multicellular organisms comprise an orderly and controllable collection of cells. The maintenance of such multicellular organisms depends on not only material and energy metabolism but also intercellular communication and signal regulation. In general, different communication signals regulate various life activities and cellular behaviours. PI3K/AKT/mTOR signalling constitutes an important pathway that consists of two parts: phosphatidylinositol 3-kinase (PI3K) and its downstream molecule serine/threonine protein kinase B (PKB; also known as AKT) [1, 2]. The PI3K/AKT/mTOR pathway is stimulated by RTK and cytokine receptor activation. Tyrosine residues are then phosphorylated and provide anchor sites for PI3K translocation to the membrane, thus participating in the transduction of various extracellular matrix molecules and cytokines [3–5]. This signalling pathway also has important biological effects on cells, such as improving viability and inhibiting senescence, ageing and death [2, 6–8], and is associated with normal and abnormal physiological activity. Dysfunction of this pathway is related to not only the occurrence and development of tumours but also many other human diseases, such as leukaemia, diabetes, and schizophrenia [9–11]. Researchers have gradually gained a strong understanding of PI3K/AKT/mTOR signalling pathway regulation and function and agree that thoroughly elucidating the mechanism of PI3K/AKT/mTOR signal transmission and the related upstream and downstream molecules is necessary [12–14]. Such knowledge will help facilitate the use of this pathway as a target for treating tumours and other related diseases. However, because the structure and function of the PI3K/AKT/mTOR signalling pathway and its relationship with upstream and downstream molecules are complex, further research is needed for a complete understanding. This review aims to summarize the recent research progress on the PI3K/AKT/mTOR signalling pathway in common human diseases (neurodegenerative diseases and tumours) and to provide a valuable reference for further research.

The article "Roles of the PI3K/AKT/mTOR signalling pathways in neurodegenerative diseases and tumours" was retracted in 2021. Reason: plagiarism.

### The PI3K/AKT/mTOR signalling pathway and its composition

The PI3K/AKT/mTOR signalling pathway consists of two parts: PI3K and its downstream molecule PKB/AKT [15] (Fig. 1).

**Fig. 1:** Overview of the PI3K/AKT/mTOR signalling pathway

#### PI3Ks

Phosphatidylinositol-3-kinases (PI3Ks) can be divided into three subtypes according to their structures and substrate specificities: class I, class II and class III. Among these kinases, the most widely studied are class I PI3Ks, which can be activated directly by cell surface receptors. Class I PI3Ks are further divided into class IA and IB based on their mode of activation. Class IA PI3Ks are activated by RTKs, G protein-coupled receptors and the small G protein RAS. On the other hand, class IB PI3Ks, which consist of only one subunit (PI3Kγ), are activated by only G protein-coupled receptors. Class I PI3Ks are composed of regulatory (p85α, p85β and p85γ) and catalytic (p110α, p110β, p110δ, and p110γ); among them, p110α and p110β are widely expressed in many tissues, while p110δ and p110γ are mainly expressed in leukocytes [12, 16]. Activation by ligands, including growth factors, results in the tyrosine phosphorylation of cell surface receptors. The p85 regulatory subunit of class IA PI3Ks binds directly to tyrosine receptors on cell membranes activated by ligands such as platelet-like growth factor and receptor-associated proteins (such as IRS1). This binding consequently activates the p110 catalytic subunit, which catalyses the conversion of PIP2 to PIP3. As a second messenger, PIP3 regulates many downstream signalling pathways. Class IB PI3Ks are heterodimers consisting of the p101 regulatory subunit and the p110γ catalytic subunit. Class IB PI3Ks are activated via the direct binding of p110γ to the Gβγ subunit of G protein-coupled receptors [15, 17, 18].

The article "Roles of the PI3K/AKT/mTOR signalling pathways in neurodegenerative diseases and tumours" was retracted in 2021. Reason: plagiarism.

Although PI3Ks play an important role in cell growth, survival, differentiation, glucose transport and metabolism, the specific mechanisms of their subunits remain unknown. In general, the important roles of the p85 catalytic and p110 regulatory subunits of PI3Ks in regulating glycolipid metabolism have been revealed by gene knockout and other approaches. For example, p110α- and p110β-knockout mouse embryos die during early development, suggesting that these two subunits have an important function in embryonic development [19]. In addition, heterozygous p110α ± or p110β ± mice do not exhibit decreased insulin sensitivity or obviously abnormal glucose metabolism. However, heterozygous mice with double knockout of these two genes show significantly impaired glucose tolerance, decreased insulin sensitivity and hyperinsulinaemia, suggesting that the two subunits play overlapping roles in the process of glycometabolism [20].

#### AKT

As the main molecule downstream of the PI3K signalling pathway, the serine/threonine protein kinase AKT comprises three subtypes, AKT1, AKT2 and AKT3, which are encoded by PKBα, PKBβ and PKBγ, respectively [3, 21]. AKT1 is widely expressed in many tissues, AKT2 is expressed in mainly insulin-sensitive tissues and at low levels in other tissues, and AKT3 is expressed in only the brain and testis. The specific tissue expression patterns of the different AKT subtypes suggest their key roles in the maintenance of physiological functions in different tissues or organs [22, 23].

The three AKT subtypes exhibit 85% amino acid sequence homology and very similar three-dimensional structures, which are composed of three different functional domains. The N-terminal pleckstrin homology (PH) domain regulates protein–protein and protein-lipid interactions. The central kinase catalytic domain is highly homologous with the regions of protein kinase A (PKA) and protein kinase C (PKC) that are responsible for enzymatic activity. Furthermore, phosphorylation of Thr308, located in this domain, is necessary for AKT activation. The regulatory region of the C-terminal AKT domain contains Ser473, which is necessary for complete AKT activation [21, 24, 25].

The article "Roles of the PI3K/AKT/mTOR signalling pathways in neurodegenerative diseases and tumours" was retracted in 2021. Reason: plagiarism.

AKT is regulated by a variety of hormones, including insulin and growth factors [26]. As mentioned above, after the PI3K regulatory subunit binds to the corresponding receptors or receptor-binding protein on the cell membrane, its catalytic subunit is activated and catalyses the formation of PIP3, which then recruits PDK1 and AKT to the cell membrane [26, 27].

PDK1 is phosphorylated at Thr308 in the AKT kinase catalytic region; PDK2 is then phosphorylated at Ser473 in the regulatory region [21]. Recent research has identified a series of potential PDK2 kinases, including integrin-linked kinase (ILK), PKCβII), DNA-dependent protein kinase (DNA-PK), mammalian target of rapamycin (mTOR) complex 2 (mTORC2) and AKT [25, 28]. Activated AKT mediates the regulation of cell growth, proliferation, the cell cycle and glycometabolism by further phosphorylating the GSK-3, FoxOs, Bad, Caspase 9, nuclear transcription factor-kappa B (NF-kappa B), mTOR and p21 proteins [25, 29].

#### AKT target proteins

##### FoxO1

The Forkhead family is a relatively new transcription factor family that was formally named in 2000 [30]. Since the discovery of the first Forkhead gene in *Drosophila* in 1989, more than 100 members of the family have been identified [31]. The common feature of the Forkhead family is a conserved DNA-binding domain called Fox, which consists of three α-helices, three β-sheets and two loops that are referred to as wings [32, 33]. Because of this feature, these transcription factors are called Forkhead/winged helix transcription factors. The Forkhead transcription factor family is currently divided into 17 subfamilies (named FoxA to FoxQ), the members of which have a wide range of biological functions [34, 35]. Among these subfamilies, the Forkhead box O (FoxO) family is the most thoroughly studied. Four distinct genes encode FoxO proteins in mammalian cells: FoxO1 (FKHR), FoxO3 (FKHRL1), FoxO4 (Afx) and FoxO6. The four homologous FoxO genes in humans are FoxO1, FoxO2, FoxO3a and FoxO4 [34]. FoxO functions in phosphorylation and acetylation posttranscriptional modifications at serine, threonine and lysine residues [35, 36]. Moreover, members of the FoxO subfamily shuttle from the cytoplasm to the nucleus and play an important role in cell proliferation, apoptosis, differentiation and oxidative stress resistance [35, 36]. As the expression level and activity of FoxO1 are significantly increased in the liver tissues of patients with severe fatty liver disease and type 2 diabetes mellitus, FoxO1 has an important role in the occurrence and progression of human metabolic syndrome [37–40]. Moreover, FoxO1 is located at the intersection of many signal transduction pathways and may become a target for the treatment or intervention of many diseases [36, 41, 42].

The article "Roles of the PI3K/AKT/mTOR signalling pathways in neurodegenerative diseases and tumours" was retracted in 2021. Reason: plagiarism.

##### GSK-3

Glycogen synthase kinase-3 (GSK-3), an important molecule downstream of AKT, is a serine/threonine protease composed of an axis inhibition protein (Axin), β-catenin and adenomatous colonic polyposis protein [43, 44]. Two GSK-3 subtypes exist: GSK-3alpha and GSK-3beta. The catalytically active regions of these two subtypes exhibit 97% sequence homology. Furthermore, GSK-3alpha and GSK-3beta are widely expressed in cells and tissues and have similar biological characteristics [45]. Recent studies have found that GSK-3beta can phosphorylate many endogenous substrates, including numerous proteins and transcription factors involved in metabolism. Therefore, GSK-3beta plays a crucial role in cell growth, development, tumorigenesis and blood sugar homeostatic regulation [43, 46, 47]. GSK-3 maintains the serine phosphorylation of IRS-1 in cells at rest and inhibits the activity of the protein. Additionally, Dokken et al. [48] reported that GSK-3 inhibits glycogen synthesis by phosphorylating glycogen synthase. Therefore, AKT can inhibit GSK-3 activity through phosphorylation and by increasing glycogen synthase activity, promoting glucose cellular uptake and glycogen synthesis, and reducing blood sugar levels. Furthermore, Lochhead et al. confirmed that GSK-3 affects the gene expression of PEPCK and G6P in the gluconeogenesis pathway [49]. GSK-3beta-knockout mouse embryos reportedly die of hepatic failure due to TNF-alpha toxicity on days 13.5–14.5 of pregnancy. However, GSK-3alpha cannot compensate for this defect, suggesting functional differences between the two GSK subtypes [50]. In pancreatic beta cells, GSK-3beta knockdown demonstrated a protective effect on apoptosis induced by endoplasmic reticulum stress [51, 52]. Moreover, GSK-3 participates in the regulation of glycogen metabolism by mediating glycogen synthesis, glucose transport, liver gluconeogenesis and beta cell function [53, 54].

##### mTOR

mTOR, a serine/threonine protein kinase, is a member of the PI3K-associated kinase protein family that participates in sensing nutritional signals and regulating cell growth and proliferation [55]. mTOR includes mTOR complex 1 (mTORC1) and mTOR complex 2 (mTORC2). mTORC1, which is composed of mTOR, Raptor and mLST8, mainly regulates cell growth and energy metabolism and is sensitive to rapamycin. mTORC2, which is composed of mTOR, Rictor, Sin1 and mLST1, is mainly involved in reconstruction of the cytoskeleton and cell survival and is not sensitive to rapamycin [56, 57]. mTORC1 is a downstream molecule of AKT and is activated by phosphorylated AKT. As a PDK2, mTORC2 fully activates AKT by phosphorylating Ser473 [58]. The AKT/TSC1–TSC2 signalling pathway can also regulate mTOR activity as well as cell growth and proliferation. TSC2 has GTPase activity and inhibits the small GTPase Rheb, which is necessary for mTORC1 activation [59]. Following phosphorylation of TSC2 by AKT, TSC2 loses its ability to inhibit mTORC1 and activate mTOR. In addition, TSC2 can be directly activated by AMPK phosphorylation, and AKT can completely inhibit TSC2 and activate mTOR by inhibiting AMPK [59, 60].

The article "Roles of the PI3K/AKT/mTOR signalling pathways in neurodegenerative diseases and tumours" was retracted in 2021. Reason: plagiarism.

The downstream effectors of mTOR include two signalling pathways, namely, 4EBP1 and S6Ks.MTOR may phosphorylate its downstream target proteins 4EBPs, and eIF4E is a subunit of the eukaryotic translation initiation complex [61]. Since hypophosphorylated 4E-BPs have a high affinity for eIF4E, phosphorylated 4E-BPs can be separated from eIF4E. The highly phosphorylated 4E-BP1 can release eIF4E, which promotes the binding of eIF4G to eIF4E to initiate the translation of relevant mRNAs [62]. Studies have shown that 4E-BPs are major regulators of mTORC1 and affect mitochondrial biosynthesis and function. In normal cells, inhibition of mTOR reduced the protein levels of ATP5O and TFAM and affected the mitochondrial DNA content, mitochondrial mass and cellular ATP levels. In 4E-BP1/2-deficient cells, mTOR did not significantly inhibit ATP5O or TFAM, but the effects of mTOR inhibition on mitochondrial biosynthesis and ATP levels were attenuated.

S6Ks proteins are another target downstream of the mTOR pathway that are encoded by two cellular genes: S6K1 and S6K2 [63]. Many studies have shown that S6K1 can affect cell growth and proliferation by promoting the translation of related mRNAs. S6K1 can directly phosphorylate relevant components and factors associated with translation mechanism, such as ribosomal protein S6, eIF4B and PDCD4 [64]. Studies have shown that mTORC1 can activate SREBP1 through S6K1 [63]. Furthermore, overactivation of mTOR enhances lipid anabolism in mouse models of obesity and diabetes. Therefore, S6Ks are the main regulators of mTOR and affect cell lipid production [65].

### Pten

The PI3K/AKT/mTOR signal transduction pathway is controlled by many factors. The tumour suppressor PTEN catalyses the reaction opposite of PIP3 generation by converting PIP3 to PIP2 [66, 67]. PTEN downregulates the PI3K/AKT/mTOR pathway to suppress cell proliferation and interfere with cellular metabolism, and inhibition of PTEN activity activates AKT and downstream pathways [68]. PTEN-knockout mice died during development due to the abnormal proliferation of various tissues. Furthermore, PIP3 levels were significantly higher in these tissues than in wild-type mice, and AKT was continuously activated [69]. Although PTEN-heterozygous mice survived, spontaneous tumours occurred. Furthermore, when PTEN was specifically knocked out in beta cells, the number and volume of these cells in mice increased significantly and induced hypoglycaemia [70, 71]. In conclusion, studies have shown that PTEN plays an important role in regulating glucose homeostasis by modulating AKT activity.

The article "Roles of the PI3K/AKT/mTOR signalling pathways in neurodegenerative diseases and tumours" was retracted in 2021. Reason: plagiarism.

### PI3K/AKT/mTOR inhibitors

Many drugs targeting single PI3K, AKT or mTOR signalling proteins (single inhibitors) or targeting both PI3K and mTOR signalling proteins (dual inhibitors) have been developed and applied in preclinical studies and cancer clinical trials. Inhibitors targeting the PI3K/PI3K signalling pathway are hoped to improve the therapeutic effect of cancer treatment. Several inhibitors that have been studied more frequently are described below (Table 1).

**Table 1:** PI3K, AKT, and mTOR inhibitors selected for preclinical and clinical development(main PI3K/AKT/mTOR inhibitors in clinical trials) [73–81]

Inhibitor	Compound or drug	Targets	Tumor types currently under investigation
PI3K	LY294002	Pan-class I PI3K	Advanced solid tumors
	Buparlisib (BKM120)	Pan-class I PI3K	Advanced solid tumors
	SAR245408 (XL-147)	Pan-class I PI3K	Advanced solid tumors
	Sonolisib (PX-866)	P110-Delta, gamma	Phase II and III trials in NHL and CLL are underway, both alone and in combination with hantiCD20 antibodies
	Pictilisib (GDC-0941)	P110-alpha, Delta	Added alpha specificity may provide benefit in MCLandsome others versus delta-only inhibitors
	Taselisib (GDC-0032)	P110-alpha, Delta	Advanced solid tumors and metastatic breast cancer (ERþ)
AKT	Pirifosine	AKT	Advanced solid tumors, multiple myeloma
	Palomid529(P529)	AKT	Advanced solid tumors, breast cancer, cervical cancer, endometrial cancer, leukemias, melanoma, multiple myeloma
	GSK2141795	AKT	Advanced solid tumors, breast cancer, cervical cancer, endometrial cancer, leukemias, melanoma, multiple myeloma
	MK-2206	AKT	Advanced solid tumors, breast cancer, colorectal cancer, endometrial cancer, head & neck cancer, lung cancer, lymphomas, pancreatic cancer, prostate cancer
mTOR	Everolimus(RAD001)	mTORC1	Approved for the treatment of renal cell carcinoma, subependymal giant cell astrocytoma associated with tuberous sclerosis, pancreatic neuroendocrine tumors, and ERþ breast cancer
	Temsirolimus	mTORC1	Approved for the treatment of renal cell carcinoma
	Rapamycin	mTORC1	Advanced solid tumors, multiple myeloma
Dual	NVP-BEZ235 (BEZ-235)	P110, mTORC1/2	Advanced solid tumors, multiple myeloma
	SAR245409(XL765)	PI3K/mTOR	Advanced solid tumors, CLL, indolent non-Hodgkin lymphoma, mantle cell lymphoma, ovarian cancer
	GDC-0980	PI3K/mTOR	Solid cancers, non-Hodgkin lymphoma, breast cancer, prostate cancer

The article "Roles of the PI3K/AKT/mTOR signalling pathways in neurodegenerative diseases and tumours" was retracted in 2021. Reason: plagiarism.

#### PI3K inhibitors

LY294002 and wortmannin are well-studied first-generation pan-PI3K inhibitors [72]. LY294002 is a reversible pan-PI3K inhibitor, and wortmannin is an irreversible pan-PI3K inhibitor. LY294002 is the first synthetic microparticle that can inhibit PI3K alpha/beta/gamma and hinder the formation of autophagosomes [73]. LY294002 sensitizes cancer cells to ionizing radiation by inactivating PKB, leading to cell cycle arrest. Because of its insolubility, short half-life, numerous nontarget effects, and unacceptable toxic effects in animal studies, its clinical application is limited. A new generation of PI3K inhibitors (including BKM120, XL147, px-866, gdc-0941 and gdc-0032) have been developed and entered clinical trials, and the representative drug is BKM120 [74]. Nvp-BKM120 (BKM120) has been shown to actively inhibit cancer cell proliferation and induce apoptosis in preclinical studies [75]. Phase I trials have shown that BKM120 is effective and well tolerated in patients with advanced cancer, and phase II and III trials are still ongoing [75].

#### AKT inhibitors

Because AKT is a key transmitter of the PI3K/AKT signalling pathway, AKT inhibitors have considerable prospects for targeted cancer therapy. Here, two well-studied AKT inhibitors, Palomid529 (P529) and Pirifosine, are mainly introduced. Palomid529 (P529) is a novel and effective AKT inhibitor that exhibits no toxicity in vivo [76]. P529 combined with radiotherapy (RT) can reportedly improve the radiosensitivity of tumour cells and induce more apoptosis and DNA double-strand breaks (DSBs), leading to delayed tumour cell growth [76]. Pirifosine, an oral alkylphosphocholine analogue, is also an effective AKT inhibitor and has shown antitumour and radiosensitivity effects in preclinical studies. Studies have reported that Pirifosine enhances the radiosensitivity of cancer cells and inhibits the phosphorylation of AKT [77] These data provide strong support for the clinical application of AKT inhibitors.

#### mTOR inhibitors

MTOR is an established therapeutic target, and rapamycin is the representative mTOR inhibitor drug. Rapamycin (sirolimus), produced by Streptococcus, was initially used as an immunosuppressant to prevent organ transplant rejection [78]. Since elucidation of the important role of mTOR in tumorigenesis and progression, it is now being studied as a tumour suppressor. Rapamycin binds to the immunosuppressive protein fkbp-12 to form an immunosuppressive complex, inhibiting the transition of mTOR and G1 to S phase transition [79]. RAD001, also known as everolimus, is a novel rapamycin derivative similar to a mTOR inhibitor that inhibits mTORC1 but has no effect on mTORC2 [80]. This drug is well tolerated and has strong antitumour properties, indicating its great prospects in cancer treatment. Rapamycin and RAD001, as well as other tacrolimus drugs, have serious side effects, such as dyslipidaemia, pulmonary toxicity and nephrotoxicity. Thus, the results of preclinical trials and early studies on mTOR inhibitors are not ideal.

The article "Roles of the PI3K/AKT/mTOR signalling pathways in neurodegenerative diseases and tumours" was retracted in 2021. Reason: plagiarism.

#### Dual PI3K/AKT/mTOR inhibitors

Short-term treatment with rapamycin and its analogues was shown to inhibit mTORC1 activity but triggered negative feedback to enhance AKT activation. On the other hand, mTOR remains activated in cancer cells even when the activities of PI3K and AKT are inhibited [78]. These disturbances and feedback between mTOR and PI3K largely limit the therapeutic efficacy of mTOR, AKT and PI3K inhibitors. Therefore, dual PI3K/AKT/mTOR inhibitors, such as BEZ235 and gdc-0980, are attracting increasing attention from researchers. BEZ235 is the first dual PI3K/mTOR inhibitor to enter clinical trials, the results of which show that the drug is well tolerated and has strong antitumour activity and is thus of substantial value for tumour treatment [81].

Studies on the PI3K/AKT signalling pathway as a targeted cancer therapy have been performed for more than a decade, and the Federal Drug Administration (FDA) has approved p110delta inhibitors for the treatment of certain types of lymphoma, providing hope for cancer treatment. A variety of PI3K/AKT signalling pathway inhibitors have been developed, but the drugs used in the clinic are limited due to the poor tolerance of patients and serious toxic side effects. Therefore, new PI3K/AKT/mTOR signalling pathway inhibitors should be developed in the future that are more effective, less toxic and more tolerable to enhance the treatment of cancer patients.

### Roles of the PI3K/AKT/mTOR signalling pathway in neurodegenerative diseases and tumours

#### Progress in understanding the role of PI3K/AKT/mTOR in AD

Alzheimer’s disease(AD), the clinical features of which include memory impairment, agnosia, visual-spatial skill impairment, executive dysfunction, and personality and behavioural changes, is the most important neurodegenerative disease [82]. The neuropathological features of AD include mainly neuronal and synaptic damage [83]. The Tau protein is essential for microtubule assembly and structural integrity maintenance, but abnormal Tau overphosphorylation and aggregation in AD lead to microtubule network instability and neurofibrillary tangle (NFT) formation, resulting in neuronal death and senile plaques [84].

The article "Roles of the PI3K/AKT/mTOR signalling pathways in neurodegenerative diseases and tumours" was retracted in 2021. Reason: plagiarism.

AKT mediates Thr212 and Ser214 phosphorylation of the Tau protein, a process catalysed mainly by PI3K-PDK1. Increased membrane levels of PIP3, the second messenger in the PI3K pathway, lead to colocalization of AKT and PDK1, which contains a PH domain, thus activating kinase-mediated phosphorylation [85]. Activated PI3K induces AKT activation and phosphorylates and inhibits GSK-3beta (GSK-3 is a multipotent serine/threonine protein kinase, and the GSK-3beta subtype has an important role in promoting Tau phosphorylation) [86]. Therefore, PI3K/AKT/mTOR signalling disorder can increase GSK-3beta activity and lead to Tau hyperphosphorylation, inducing NFT formation [87, 88]. This finding also explains the observed PI3K/AKT/mTOR signal attenuation in the brains of AD patients.

The amyloid beta (Ab) protein (the main component of precipitated plaques) also interacts with the PI3K/AKT/mTOR pathway [89]. Abeta induces neurotoxicity by inhibiting the PI3K/AKT/mTOR pathway in neuronal cells and neural stem cells. GSK-3beta is mainly activated by Abeta oligomers, blocking PI3K/AKT/mTOR pathway activity, which increases Tau protein hyperphosphorylation [90].

#### Progress in understanding the role of PI3K/AKT/mTOR in PD

Parkinson’s disease (PD), one of the most common neurodegenerative diseases, involves many motor symptoms (such as quiescent tremors, rigidity, and postural instability) and nonmotor symptoms (such as autonomic nervous, mental, sensory, and cognitive impairments) [82]. Despite the many studies on PD over the years, its pathogenesis remains unclear, and treatment remains difficult [91]. Studies have shown that AKT also plays a role in PD signal transduction. As serine/threonine-specific protein kinases, AKT and phosphorylated AKT are significantly reduced in the substantia nigra pars compacta (SNpc) of PD patients [92]. PI3K/AKT/mTOR pathway activation also promotes the survival and growth of dopamine neurons by inhibiting apoptosis, thus preventing PD [93]. Experiments have shown that AKT can inhibit the activity of GSK-3 by phosphorylating Ser21 of GSK-3alpha or Ser9 of GSK-3beta. Moreover, abnormal regulation of GSK-3beta can lead to the pathophysiological manifestations of PD. Some studies have suggested that GSK-3beta is abnormally expressed in PD [94–96].

The article "Roles of the PI3K/AKT/mTOR signalling pathways in neurodegenerative diseases and tumours" was retracted in 2021. Reason: plagiarism.

The PI3K/AKT/mTOR pathway affects the oxidative stress pathway through other downstream signalling molecules, such as FoxO3a, in addition to regulating GSK-3beta to influence PD. In the case of abnormal Parkin gene expression, oxidative stress becomes imbalanced primarily because the PI3K/AKT/FoxO3a pathway is disrupted, leading to PD [97]. The levels of mTOR, a downstream signalling molecule in the PI3K/AKT/mTOR pathway, were also found to be significantly reduced in the brain tissues of PD patients, although the PI3K/AKT/mTOR pathway was found to have a protective effect on neurons [98]. Therefore, PI3K/AKT/mTOR affects PD largely by influencing downstream signalling molecules that regulate apoptosis.

The PI3K/AKT/mTOR signalling pathway can affect signal regulation in PD patients by modulating downstream protein molecular targets, such as GSK-3beta, mTOR and FoxO3a. Researchers have also begun to study potential drugs to treat PD, including salidroside (SAL), which can suppress GSK-3beta through the PI3K/AKT/mTOR pathway and thus reduce PD symptoms [99].

#### Research progress on PI3K/AKT/mTOR in HD

Early Huntington’s disease (HD) often manifests as irregular muscle twitches, such as finger flexion and extension, nodding and facial muscle twitching. HD symptoms further develop into sudden, purposeless and intense involuntary dance-like movements of the face, neck, limbs and trunk, followed by corresponding psychiatric symptoms, such as depressive mood disorder and various degrees of personality changes [100].

Inhibition of any part of the RAS/PI3K/AKT pathway significantly reduces the survival of cultured sympathetic neurons in the presence of nerve growth factor (NGF). As an upstream factor, RAS inhibits apoptosis through PI3K, indicating that the PI3K pathway is key for cell survival and neuron protection [101]. Brain-derived neurotrophic factor (BDNF), which regulates neurotransmitters, also plays an important role in the survival and growth of neurons, contributing to their plasticity, and is an indispensable cytokine for learning and memory. Some studies have shown that BDNF can bind to tropomyosin receptor kinase B (Trkb) and activate the PI3K/AKT pathway, thus protecting neurons and preventing HD development [102].

Furthermore, the Tau protein is substantially hyperphosphorylated in HD neurons, serving as a pathological manifestation of HD [103]. Studies have shown that GSK-3beta, which is downstream of PI3K/AKT, is a crucial factor leading to Tau protein hyperphosphorylation and is reversely regulated by the PI3K/AKT pathway. Therefore, PI3K/AKT signalling also regulates Tau protein hyperphosphorylation through the downstream molecule GSK-3beta and participates in the occurrence and development of HD [104].

The article "Roles of the PI3K/AKT/mTOR signalling pathways in neurodegenerative diseases and tumours" was retracted in 2021. Reason: plagiarism.

In summary, the PI3K/AKT signalling pathway is involved in the occurrence and development of various neurodegenerative diseases, with important functions in the proliferation of cells, inhibition of apoptosis and oxidative stress and regulation of a variety of downstream molecules. The PI3K/AKT pathway is also associated with many other pathways. In general, the study of PI3K/AKT pathway molecules and their interactions will provide new ideas for the mechanistic analysis of neurodegenerative diseases and corresponding drug development.

#### Research progress on the PI3K/AKT/mTOR signalling pathway in cancer

The occurrence and development of malignant tumours are the result of interactions between multiple signal transduction pathways. The PI3K/AKT/mTOR signal transduction pathway is abnormally activated in many tumorigenesis processes and has a key role in tumorigenesis and development. Furthermore, the PI3K/AKT/mTOR pathway is involved in regulating the survival, proliferation, invasion and migration of cancer cells. Accordingly, inhibition of this pathway has become a hot research topic in cancer therapy.

##### Role in promoting tumorigenesis

The PI3K/AKT/mTOR signalling pathway participates in cell cycle processes and promotes the occurrence and development of tumours. Many downstream molecules constitute the PI3K/AKT/mTOR signalling pathway, such as mTOR, and activated AKT directly phosphorylates and thus activates mTOR. mTOR then promotes the binding of cyclin D1 to cyclin-dependent kinase (CDK) to initiate cell division. High levels of cyclin D1 expression can induce cell cycle transition from the G1 to S phase, shorten the cell cycle and accelerate cancer development. P27kip1 belongs to the CDK inhibitor protein family and negatively regulates the cell cycle; it inhibits the activity of CDK, leading to cell cycle arrest and blockage of cell proliferation. AKT inhibits the cell cycle blockade by phosphorylating P27kip1 and accelerates cell proliferation and differentiation [105]. Additionally, mTOR helps to regulate the synthesis of biological macromolecules such as proteins, nucleotides, and lipids, thus providing the materials necessary for cancer cell growth [106].

##### Role in controlling angiogenesis

Angiogenesis is the basis of the growth, metastasis and lethality of tumours. The PI3K/AKT/mTOR signalling pathway is not only involved in regulating the proliferation and apoptosis of cancer cells but is also closely related to angiogenesis; moreover, the PI3K/AKT/mTOR pathway promotes normal and tumour angiogenesis [107]. Activated AKT causes eNOS distribution in the vascular endothelium by phosphorylating Ser1177, resulting in nitric oxide (NO) production in blood vessels. This phenomenon helps to regulate vascular function and causes vasodilation, vascular remodelling and angiogenesis [108]. In addition, AKT activation induces the expression of high levels of HIF-1, an important regulator of angiogenesis that can upregulate the expression of VEGF and other angiogenic factors, thereby promoting angiogenesis. HIF-1 affects vascular endothelial cells through the following mechanisms of action: (1) promoting the migration and proliferation of endothelial cells; (2) increasing vascular permeability, plasma protein exosmosis, and cellulose scaffold formation to help vascular endothelial cells migrate and provide support for vascular growth; and (3) activating the proteolytic enzyme system, degrading the extracellular matrix and promoting angiogenesis [109–112].

The article "Roles of the PI3K/AKT/mTOR signalling pathways in neurodegenerative diseases and tumours" was retracted in 2021. Reason: plagiarism.

##### Role in promoting cancer cell invasion and metastasis

The PI3K/AKT/mTOR signalling pathway plays an important role in promoting tumour invasion and metastasis via the following mechanisms. (1) Activated AKT enhances the transcriptional activity of NF-kappa B, promotes the transport of tumours, and supports the invasion of tumours. (2) Actin polarization is promoted, and AKT1, a downstream molecule of PI3K, is reportedly involved in regulating the invasion and metastasis of breast cancer cells. Palladin is an actin-related protein that participates in cytoskeleton construction, regulates the structure of the actin system and importantly functions in cell migration. AKT1 can phosphorylate Ser507 of palladin to regulate the invasion and metastasis of cancer cells [113]. (3) Activation of matrix metalloproteinases (MMPs), a group of proteolytic enzymes that participate in degrading the extracellular matrix, promotes cell invasion and metastasis. There are 23 types of MMPs, and MMP-2 and MMP-9 are known to be crucial for cell invasion. PI3K/AKT/mTOR can promote the expression of MMP-2 at the mRNA and protein levels, degrade the extracellular matrix, and promote the invasion and metastasis of cancer cells [106].

Based on the above findings, the PI3K/AKT/mTOR pathway plays an important role in tumorigenesis and development. When stimulated by upstream signals such as growth factors, PI3K activates AKT, which further activates downstream signalling molecules and regulates cancer cell proliferation, invasion and metastasis, angiogenesis, and carbohydrate metabolism. Accordingly, the growth and metastasis of tumours can be inhibited by suppressing the expression of each molecule in the pathway and blocking signalling, resulting in an antitumour effect. The development of targeted drugs following an in-depth study of the PI3K/AKT/mTOR signalling pathway is of great significance for cancer treatment.

The article "Roles of the PI3K/AKT/mTOR signalling pathways in neurodegenerative diseases and tumours" was retracted in 2021. Reason: plagiarism.

## Perspectives

The PI3K/AKT/mTOR signalling pathway is an important signal transduction pathway that has many biological functions and is mediated by enzyme-linked receptors in mammals [114]. This pathway regulates biological activity by modulating the epigenetic modification of DNA and histones of target genes and plays important roles in cell differentiation, muscle development, environmental adaptation and disease development [2, 3, 115]. PI3K/AKT/mTOR signalling components also phosphorylate and produce precursor apoptotic proteins, such as Bad. Short-term actions to prevent apoptotic pathway activation and ultimately lead to cell death have crucial roles in cell growth, proliferation and apoptosis and promote insulin-stimulated glucose uptake and storage. Overall, research on the biological activity of the PI3K-AKT pathway establishes an indispensable link between the growth and development of organisms and metabolism. PI3K/AKT/mTOR cascades in different cells produce different physiological and pathological effects that can lead to different pathophysiologies.

In conclusion, a thorough understanding of the key regulatory steps of the PI3K/AKT/mTOR pathway in various human diseases will help to elucidate the pathogenesis of cerebrovascular diseases, neurodegenerative diseases, diabetes mellitus and malignant tumours. More importantly, such research can provide new molecular targets (such as biological markers and genetic diagnoses) for the diagnosis and treatment of human diseases.

## Data Availability

Not applicable.
